# The Use of Big Data Combined with Artificial Intelligence Neural Network Technology in Urban Spatial Evaluation System

**DOI:** 10.1155/2022/7936522

**Published:** 2022-06-10

**Authors:** Lei Wang, Yujie Liang, Gaizhen Shang, Zhiyong Song, Peng Gao

**Affiliations:** ^1^NORENDAR International Ltd., Shijiazhuang 050011, Hebei, China; ^2^Urban and Rural Construction College, Agricultural University of Hebei, Baoding 071066, Hebei, China

## Abstract

This exploration aims to promote the development of urbanization in China and improve the utilization rate of urban resources. First, intensive theory and spatial economics are studied. Next, an input-output urban spatial evaluation system is established based on intensive theory and data envelopment analysis (DEA). Then, deep learning (DL) is adopted for optimization, and an urban space evaluation system based on DL is proposed. Finally, the reliability level of the urban space evaluation system is tested. The results show that the model's input and output index *α* values are above 0.9, and the overall reliability level is higher than 0.9, indicating that the urban space evaluation system has a high reliability. The training results of the DL model show that the mean absolute error (MAE) of model prediction decreases gradually with the increase of training time and training times. When the training lasts for 5 min, each index' MAE is basically stable between 0.22 and 0.23, and the evaluation accuracy is obvious. The urban space evaluation system based on DL has higher evaluation accuracy, reaching 83.40%. Therefore, this exploration can provide research experience for promoting the effective utilization of urban resources and provide a reference for formulating an urbanization evaluation index system suitable for China's national conditions.

## 1. Introduction

Data mining, machine learning, and artificial intelligence (AI) technology rise with the continuous progress of big data technology, which has brought breakthroughs to the development of science and technology [1]. In 2015, the State Council issued the Action Platform for Promoting the Development of Big Data, which proposed to promote the development and application of big data, accelerate the government's data sharing, and make an overall plan for the construction of big data infrastructure [2]. The Outline of the 13th Five-Year Plan for National Economic and Social Development of People's Republic of China issued in March 2016 proposed to take big data as a primary strategic resource to promote the development of big data comprehensively [3]. With its large-scale, high coverage, and quantitative characteristics, big data has become an indispensable strategic resource for all walks of life in China and has also had a great impact on the urban and rural planning industry. Therefore, big data has become an important tool to assist all aspects of urban planning and promote the development of smart cities in China.

The evaluation of urban development level is conducive to improving urban development speed. Scholars have done a lot of research to evaluate the city's development status and future potential. Ye (2019) established an evaluation indicator system for urban development quality from six aspects: science and technology, education level, government management, resources and environment, openness, and infrastructure. Moreover, the methods of entropy analysis and cluster analysis were used to make an empirical analysis on the urban development of Guangdong Province, and corresponding suggestions were put forward [4]. Navarro-Yáñez et al. (2020) used the plan quality evaluation method to analyze the quality of local plans formulated under the European policy framework of Spain and the factors explaining the quality level of these local plans. The scale to measure the plan quality was proposed based on the five main dimensions (factual basis, objectives, policy actions, plan governance, and evaluation) [5]. Basile et al. (2021) studied and analyzed the economic spatial structure and considered that economy was an interconnected multilayer structure with spatial dimension, and the spatial distribution of economic activities evolved into a complex model over time [6]. Shen et al. (2021) established a consistency measurement framework to reveal how planning affected substandard urban development. The multi-indicator framework included quantitative indicators, the spatial distribution relationship between urban new unqualified land and zoning map, the location of urban new unqualified land, and the original land use [7]. Parivar et al. (2021) adopted the evaluation framework composed of three dimensions and 16 indicators based on the conceptual principle of the close relationship between structure and function and analyzed the development of Yazd in Iran using the analytic hierarchy process [8]. The research and analysis of the above scholars reveal that most present evaluation studies only stay in the evaluation stage. The index system is not established, and the evaluation model is not selected. It leads to the disconnection between evaluation and morphological optimization and greatly reduces evaluation effectiveness. Therefore, the organic integration of evaluation and morphological optimization is the right way to give full play to the effectiveness of evaluation.

In conclusion, under the trend of the rapid development of digital technology, the effective evaluation of the urban spatial system by using AI technology is of great significance to social development. Therefore, the research innovation is to establish an input-output urban spatial evaluation system based on intensive theory and data envelopment analysis (DEA) and optimize the system through deep learning (DL). The research results provide a powerful tool for understanding the current level of urban development and help to promote the efficient utilization of urban resources.

## 2. Construction and Optimization of the Urban Spatial Evaluation System

### 2.1. Intensive Theory and Spatial Economics

Intensive development is a theory involving a wide range of fields and diversified contents. It is a cross-cutting theory integrating multiple areas such as economy, technology, and ecology [9]. The concept of intensification first appeared in economic theory. In 1817, David Ricardo applied it to the land tax theory in Political Economics and Tax Principles. It was proposed to use advanced technology and management methods to concentrate more means of production and labor into a small area of land to obtain a higher income [10]. Later, in 1930, Marx applied the concept of intensification to the book Das Kapital. In the agricultural economy, it was proposed that, in economics, the so-called intensive farming meant that capital was concentrated on the same land rather than scattered on several adjacent lands [11]. “Intensive operation” in the sense of modernization refers to using the lowest input to obtain the highest benefit. Its essence is to study the benefit relationship between input and output [12]. The intensive development of cities is mainly aimed at the space resource reduction and environmental pollution caused by the relatively extensive development form in China for a period. It relies on the progress of science and technology to improve the resource utilization and operation efficiency of cities and promote the intensive development of urban industries. The main indicator to measure the intensive level is the intensive degree [13]. Urban informatization, digitization, and complexity have become a great challenge for urban design in the gradual expansion of urban space. Meanwhile, they are also important opportunities for technological innovation. Unlike local space form design, intensive development can be more inclined to the perceptual cognition of visual aesthetics. In the face of more diverse urban constituent elements, the overall urban spatial form design tends to be more rational. It needs scientific and technical methods as support to assist the government decision-making departments to formulate policies in line with the urban spatial characteristics and systematic laws. Since the intensive theory is first put forward based on land management, the concept of intensive degree is also based on this theory. Intensive degree refers to the utilization rate of land per unit area, which can be measured by physical form, value form, or indicators. The equation is that

(1) $$\begin{array}{c} I=\frac{\left(A+K+Z\right)}{F}. \end{array}$$

*I* represents intensity, *A* represents labor wage, *K* represents capital consumption, *Z* represents operating capital interest, and *F* represents the operating land area.

Spatial economics [14] is an intermediate link in the transformation from structural economics to development economics. Its research objects are the spatial layout of production factors and the competitive phenomena and laws of space. The main theory is increasing returns to scale; that is, when the number of inputs increases by the same percentage, the total return will increase by a percentage greater than this percentage. Spatial economics is the internal motivation and basic law of urban development.

### 2.2. Artificial Neural Network (ANN)

ANN is an algorithm model for parallel or distributed data processing by imitating the brain's neural network and function [15]. ANN model is highly nonlinear and can deal with complex logic operations. It is full of many interrelated nodes, which can be called neurons. Neurons are the basic components of neural networks and each neuron contains a specific “output function.” Figure 1 shows its structure.

In Figure 1, *X*1, *X*2, and *X*3 on the left represent the neuron input, and *Y* on the right represents the neuron output. *W*(1,2,…, *i*) refers to the directional arc with variable weight connecting each neuron for signal transmission and processing. Multiple neurons are connected with each other to form a complex network system. A complete ANN consists of three different structural units: input layer, output layer, and hidden layer. The input layer will preliminarily process the data and signals to be processed. The data processed and received by the input layer will be output from the input layer and enter the hidden layer. The hidden layer will deeply mine the hidden information in these data and transfer the hidden information to the output layer. Usually, an ANN contains multiple hidden layers.  Figure 2 shows the structure of ANN.

### 2.3. Application Analysis of DL in Urban Spatial Evaluation

DL [16] is derived from ANN and it is proposed to distinguish it from traditional shallow learning [17]. The ability of shallow learning to represent complex functions is limited, and the generalization ability for complex classification problems is also limited. The essence of DL is to learn data features from complex big data and improve the accuracy of classification or prediction by building more hidden layers. The purpose of DL is “feature learning.” Figure 3 shows the characteristics of DL compared with shallow learning.

DL has similarities and differences with traditional neural networks. The similarities are that both are multilayer network structures composed of the input layer, hidden layer, and output layer, and only the nodes of adjacent layers are connected. The difference lies in their different training mechanisms. The traditional neural network adopts an error backpropagation training method. It means that an initial value is input into the neural network to obtain an output value. Then, the error between the output value and the standard value is calculated, the error is back-transferred, and the parameters of each layer of the neural network are corrected in turn. However, DL is basically a layer-by-layer training method.

In the DL model construction, in addition to the construction of the input layer, hidden layer, and output layer, it is also necessary to select hidden function, optimization function, loss function, and evaluation criteria. At present, the commonly used activation functions are Sigmoid (Logistic Activation Function) [18], Tanh (hyperbolic tangent function) [19], and Relu (rectified linear unit) functions [20].

The Sigmoid function can also be called the logistic function. It compresses a real number in the range of 0–1, which can change negative numbers to 0 and large positive numbers to 1. The function expression reads

(2) $$\begin{array}{c} f\left(x\right)=\frac{1}{1+e^{-x}}. \end{array}$$

Figure 4(a) is its function graph and derivative graph.

The derivative graph of the Sigmoid function shows that its graph near *x* = 0 is flat; that is, the map of the Sigmoid function near *x* = 0 is close to 0. During backpropagation, the gradient will disappear. Besides, the output of the Sigmoid function is not zero mean, and it is an exponential function with a relatively large amount of calculation.

Tanh function, also known as hyperbolic tangent function, also compresses a real value, and its function expression reads

(3) $$\begin{array}{c} \text{Tanh}\left(x\right)=\frac{\text{sinh}\left(x\right)}{\text{cosh}\left(x\right)}=\frac{e^{x}-e^{-x}}{e^{x}+e^{-x}}. \end{array}$$

Figure 4(b) is a function graph of the Tanh function and its derivative graph.

The output range of Tanh function between −1 and 1 is zero mean, but there is still the problem of gradient disappearance.

The Relu function is to perform a semicorrection from the bottom, and its function expression is

(4) $$\begin{array}{c} f\left(z\right)=\text{max}\left(0,z\right). \end{array}$$

When *z* < 0, the value of the function is 0. When *z* = 0, the function value is 0. When *z* > 0, the function value is *z*.

Figure 4(c) is a graph of the function and its derivatives.

Relu function can make the network converge faster, have no saturation, and resist the gradient disappearance. It is very efficient in calculation, but it will be very fragile in training because it changes all negative input numbers to 0. The gradient disappearance only appears when *x* < 0. Therefore, the Relu function is selected as the activation function.

Adaptive moment estimation (Adam) is used as the optimization function. It can modify the weight of neural networks iteratively based on training data.

Mean-Square Error (MSE) function is selected as the loss function, which reflects the average value of the square difference between the estimated value and the true value, and can be used to evaluate the accuracy of the experimental data. The function expression reads

(5) $$\begin{array}{c} \text{MSE}=\frac{1}{M}\sum_{m=1}^{M}{\left(y_{m}-\hat{y_{m}}\right)}^{2}. \end{array}$$

*M* represents the total number of training samples, *m* refers to the training samples, *y*_*m*_ represents the true value, and $\hat{y_{m}}$ is the predicted value.

Mean Absolute Error (MAE) function is selected as the evaluation standard. It represents the average value of the absolute error between the expected value and the true value. The function expression reads

(6) $$\begin{array}{c} \text{MAE}=\frac{1}{M}\sum_{m=1}^{M}\left|y_{m}-\hat{y_{m}}\right|. \end{array}$$

From the physical point of view, urban public space is spatial and needs to be implemented into specific spaces. However, public space attributes also include humanistic. The traditional planning big data is still static and physical. Although there is certain objectivity, the consideration of human activities in the rapidly changing urban space system is still insufficient. Only using the existing traditional data and traditional methods for analysis will lead to many public space evaluations, planning, and decisions often based on this fuzzy and uncertain logical relationship. The introduction of various neural network algorithms in DL technology can use the excellent feature extraction ability of the neural network to extract the required data independently based on intelligent data collection. It eliminates a large number of manual screening and data cleaning processes. After the introduction of the neural network, it is not necessary to consider the specific relationship between these data and the final analysis results. Only a certain amount of samples is needed for training. Then, the neural network can learn the mapping relationship between data and results and focus on exploring how to make urban public spaces better meet people's activity needs.

### 2.4. Establishment of an Urban Evaluation System Based on DEA

DEA method [21] includes operational research, management, mathematical economics, and other fields and uses a mathematical programming model to evaluate the effectiveness of the Decision-Making Unit (DMU) with multiple inputs and outputs. The efficiency of multiple service units providing similar services is compared by explicitly considering the use of multiple inputs and the generation of multiple services. DEA effectiveness can be used to judge whether the combination of input and output reaches the optimal efficiency. It is adopted to evaluate the degree of urban intensification.

Based on the DEA method, each block in the city can be regarded as a DMU unit, and the intensive urban spatial evaluation can be equivalent to calculating the DEA effectiveness of the combination of input and output elements in the street area of the city. When DEA is effective, it indicates that the street area's input-oriented elements and output-oriented elements in the evaluation city sample have reached the optimal combination. It means that, under the current block conditions, the form of the street area in the evaluation sample has reached intensification. Meanwhile, using the DEA evaluation model for comprehensive evaluation does not need to find evaluation standards, but to use the statistical methods to realize by relying on self-comparison in many data samples.

*n* represents the number of cities that need intensive evaluation. There are *m* input types and *s* output types of cities. *X*_*ij*_ represents the total amount of the *i*-th input element of the *j*-th town. *Y*_*rj*_ represents the total amount of the *r*-th output element of the *j*-th town. The input expression of the *j*-th town reads

(7) $$\begin{array}{c} X_{j}=\left(X_{1j},X_{2j},\ldots ,X_{mj}\right). \end{array}$$

*v* ^*T*^ represents the input weight coefficient, and its expression reads

(8) $$\begin{array}{c} v^{T}=\left(v_{1},v_{2},\ldots ,v_{m}\right). \end{array}$$

The output expression of the *j* -th town reads

(9) $$\begin{array}{c} Y_{j}=\left(Y_{1j},Y_{2j},\ldots ,Y_{sj}\right) \end{array}$$

*u* ^*T*^ represents the output weight coefficient, and its expression reads

(10) $$\begin{array}{c} u^{T}=\left(u_{1},u_{2},\ldots ,u_{s}\right) \end{array}$$

The efficiency evaluation indicator of the *j*-th town is

(11) $$\begin{array}{c} h_{j}=\frac{u^{T}Y_{j}}{v^{T}X_{j}}=\frac{\sum_{r=1}^{s}u_{r}Y_{rj}}{\sum_{i=1}^{m}v_{i}X_{ij}}. \end{array}$$

Anderson and Peterson proposed to introduce slack variable *s*^−^ and remaining variable *s*^+^ to optimize the DEA model in 1993. A superefficiency DEA model is proposed, and its equation is

(12) $$\begin{array}{c} \begin{array}{cc} \min, & \theta_{0},\\ \text{subject to,} & \sum_{j=1}^{n}\lambda_{j}x_{j}+s^{-}=\theta_{0}x_{0}, \end{array}\\ \sum_{j=1}^{n}\lambda_{j}y_{j}+s^{+}=y_{0}. \end{array}$$

*λ*_*j*_ ≥ 0, *j*=1,2,…, *n*, *s*^−^ ≥ 0, and *s*^+^ ≥ 0. *θ*_0_ represents the efficiency value of the evaluation unit. The model is solved. When *θ*_0_=0, *s*^−^=0, and *s*^+^=0, DEA is effective; that is, when the input is certain, its output reaches the maximum. When  *θ*_0_ < 0, *s*^−^ > 0, and *s*^+^ > 0, non-DEA is effective; that is, under a certain input, its output does not reach the maximum value.

According to the DEA model, the indicators in the urban spatial evaluation indicator system can be divided into input-oriented indicators and output-oriented indicators. The spatial morphological characteristics of cities can be described from three aspects: transportation, land use, and development.

Street integration, motor traffic capacity, and rail transit convenience can be selected to describe urban traffic.

Integration degree is the degree of dispersion between one element and other elements in space. By calculating the integration degree of streets, people can have a preliminary understanding of the convenience of urban ground transportation. The degree of integration is represented by *RA*_*i*_.

Motor traffic capacity is the capacity of cities for vehicles, and this indicator is also a main content of urban traffic planning. TV is used to represent motor traffic capacity.

Rail transit convenience mainly describes the convenience of urban underground rail transit. With the continuous development of science and technology, underground rail transit represented by the subway has gradually become the main indicator to evaluate the development of urban transportation and one of the crucial elements of urban spatial form because of its high speed and low pollution characteristics. RA is adopted to indicate rail transit convenience.

Urban land use is mainly described by building density, floor area ratio, and land structure.

Building density is used to describe the floor area of the building bottom. It is an important indicator to measure the urban land utilization rate, represented by BD.

The floor area ratio is a comprehensive indicator used to evaluate the intensity of urban land use, reflecting the overall level of urban land use efficiency.

Land use structure is mainly used to evaluate the rationality of urban land use planning and is a critical evaluation indicator of urban spatial structure. The rationality of urban land structure is evaluated by taking residential land, public management and service land, industrial land, transportation facilities land, and green land as the main land types, and the weight of each land type is 0.2. Among the five types, *LUR*_*i*_ represents the land use proportion of a single type.

*C*_*i*_ represents the land area of a single type among the five types of residential land, public management and service land, industrial land, transportation facilities land, and green space. *A* represents the total land area of urban buildings.

According to the Standard for Classification and Planning of Urban Land for Construction (GB50137–2011), Table 1 shows the standard values of five types of land.

The land use structure score is expressed by LUS, and its expression reads

(13) $$\begin{array}{c} \text{LUS}=\sum_{i=1}^{5}\left(1-\frac{\left|LUR_{i}-LUR^{\prime }{}_{i}\right|}{LUR^{\prime }{}_{i}}\right)*0.2. \end{array}$$

*LUR*_*i*_′ represents the standard value of single type land use.

Urban development is mainly described by regional coverage of public facilities, infrastructure operation efficiency, land use functional diversity, and population density.

The regional coverage rate of public facilities is to evaluate the balance degree of urban public facilities layout, expressed by CP.

Infrastructure operation efficiency refers to the operation efficiency of infrastructure required for five residential activities: water supply, power supply, gas supply, drainage, and sanitation. It is used to evaluate the operation efficiency of cities, expressed by EIO.

Land use functional diversity is an important indicator to evaluate urban spatial vitality. Land use diversity is conducive to the intensive development of cities, expressed by *D*.

Population density can reflect cities' carrying capacity and spatial vitality to a certain extent, and the calculation is simple. PD indicates population density.

Among these indicators, integration degree, motor traffic capacity, rail transit convenience, land use structure, and public facilities area coverage are input-oriented indicators, and building density, floor area ratio, infrastructure operation efficiency, land function diversity, and population density are output-oriented indicators.  Figure 5 shows the urban spatial evaluation system.

### 2.5. Optimization of Urban Spatial Evaluation Based on DL

Although DEA can be better applied in intensive evaluation, it has some limitations for different types of urban forms in practice, because it is too idealistic and absolute. Therefore, it is necessary to optimize the evaluation criteria to a certain extent according to the actual situation. Hence, DL technology is introduced to optimize the evaluation model. The development of urban spatial form is the result of the joint action of multiple factors, which have certain laws. DL model is adopted to learn these laws and then predict the spatial form of cities.

Figure 6 is a DL-based morphological optimization process.

## 3. Results

### 3.1. Reliability Test of the Urban Spatial Evaluation System

The reliability of the urban spatial evaluation system is tested through Cronbach's *α* coefficient.  Table 2 shows the results.

Table 2 shows that the *α* value of the input indicator of the constructed urban space evaluation system is 0.92, with a high reliability level, and the *α* value of the output indicator is 0.9178, also with a high reliability level. The overall reliability level is also above 0.9, indicating that the constructed indicator system meets the requirements.

### 3.2. Analysis of Model Training Results

Sample data from 587 towns in Hebei Province are used to train the DL network.  Figure 7 shows the change of MAE value of each indicator with the increase of training time.

Figure 7 shows that, with the increase of training time and model training times, the MAE value of the model becomes increasing slower and its decreasing speed is also increasing slower, until it reaches the expected value that tends to be stable. When the training lasts for 5 min, the MAE values of each indicator are between 0.22 and 0.23. The results show that, with the increase of training time and training times, the accuracy of model prediction gradually increases until it reaches the expected value.

The proposed DEA-based evaluation system is further compared with the DL-based optimization system and the algorithm proposed by Shen et al. [7] to analyze its evaluation accuracy, as shown in Figure 8.

Figure 8 shows that the evaluation accuracy of the optimization evaluation system based on the DL proposed reaches 83.40%, which is at least 2.37% higher than that of other model algorithms. It means that, after the optimization of AI technology such as DL, the average accuracy of the model algorithm of the optimized urban space evaluation system constructed is better.

## 4. Conclusion

At present, China is in an important period of rapid urbanization. Given the low efficiency of urban space in China, an input-output urban space evaluation system based on DEA is established. Moreover, the system is further optimized by using DL language, and an urban space evaluation system based on DL is constructed. Finally, the reliability level is tested and the DL model is trained. The results show that the model's value of input and output index *α* is more than 0.9, and the reliability level is high. With the increase of model training time, the MAE value of each index decreases, and the prediction accuracy of the DL model reaches 83.40%. Therefore, the model has certain practicability and can provide research experience for the subsequent improvement of urban resource utilization. However, there are still some research deficiencies. First, the output of the DL model is unstable, which will be studied in further research. Next, based on establishing a stable model, further comparison and evaluation of urban space utilization in different years is also the future research direction.

## Figures and Tables

**Figure 1:** Basic composition of neurons.

**Figure 2:** ANN structure diagram.

**Figure 3:** Characteristics of DL.

**Figure 4:** Function graph and its derivative graph: (a) Sigmoid function; (b) Tanh function; (c) Relu function.

**Figure 5:** Urban spatial evaluation indicator system (RA_i_ represents the integration degree indicator, TV represents the motor traffic capacity indicator, RA represents the rail transit convenience indicator, LUS represents the land structure scoring indicator, CP represents the regional coverage rate of public facilities, BD represents the building density indicator, FAR represents the floor area ratio, D represents the land use diversity indicator, EIO represents the infrastructure operation efficiency indicator, and PD represents the population density indicator).

**Figure 6:** DL-based optimization process.

**Figure 7:** MAE changes of urban spatial evaluation index with the increase of training time: (a) MAE changes of input indicator with the increase of training time; (b)MAE changes of output indicator with the increase of training time.

**Figure 8:** Precision comparison results of urban space evaluation system under different algorithms.

**Table 1:** Standard values of five types of land use.

Land type	Proportional standard value
Residential land	25.0%–40.0%
Public management and service land	5.0%–8.0%
Industrial land	15.0%–30.0%
Transportation facilities land	10.0%–30.0%
Green land	10.0%–15.0%

**Table 2:** Reliability test of the urban spatial evaluation system.

Indicator dimension	*α*
Input indicator dimension	0.9235
Output indicator dimension	0.9178
Total	0.9297

## Data Availability

Data are available on request.
